# Relations between entrepreneur’s social identity and strategic entrepreneurship: Sustainable leadership as mediator

**DOI:** 10.3389/fpsyg.2022.903927

**Published:** 2022-09-26

**Authors:** Gang Liu, Qing Yin, Leyi Zhang

**Affiliations:** ^1^School of Business, East China University of Science and Technology, Shanghai, China; ^2^Putra Business School, Selangor, Malaysia

**Keywords:** sustainable leadership, strategic entrepreneurship, entrepreneur’s social identity, family firm, sustainable growth

## Abstract

Although there are studies verifying that strategic entrepreneurship is positively related to the risk resistance and performance of enterprises, it is unclear how enterprises can implement effective strategic entrepreneurial activities in dynamic situations. This research aims to explore why and how the entrepreneur’s social identity influences and drives firm’s strategic entrepreneurial activities. In this study, it applied case study method to interview a technology-based family firms that have effectively conducted strategic entrepreneurial activities to meet challenges, and uses grounded theory for data analysis. The research finds that (1) the social identity of entrepreneurs actively promotes the strategic entrepreneurial activities of enterprises; (2) sustainable leadership mediates the relationship between social identity and strategic entrepreneurship; (3) at different stages of enterprise development, entrepreneurs dynamically adjust their social identity types to enhance sustainable leadership; (4) through the focus and extension of technological advantages, sustainable leadership ensures that enterprises can promote the implementation of strategic entrepreneurial behavior by disintegrating and integrating the value chain. This study explores the strategic entrepreneurship path of family firms and also provides new insights for future research on the strategic entrepreneurship and sustainable growth of such firms.

## Introduction

Family firms are owned and typically managed by family members (Shepherd and Haynie, 2009). These firms have greater liberty to act unilaterally and idiosyncratically than non-family firms, so the behavior of them is distinctively influenced by the characteristics of family owners and managers (Chrisman and Patel, 2012). Among them, one typical representative is technology-based family firms, where the family members master the advanced technologies, production processes and patents of product manufacturing. These technologies and resources can be used to produce products with excellent performance and broad market that are difficult to be imitated or surpassed by competitors in a short period of time (Rydehell, 2020).

Over the past 40 years of reform and opening up, China’s economy has undergone a transition from a planned economy to a market economy. In this process, the relationship between market and the government has undergone fundamental changes, which have had profound impacts on various economic forces, including state-owned and private firms. Technology-based family firms, as a typical representative of family firms, are purely market-based and have been growing and developing continuously with the continuous marketization of the Chinese economy. These firms are distributed in various areas such as new materials, new energy, information technology, artificial intelligence and integrated circuits, and have become an important force in promoting technological innovation, increasing employment and improving people’s livelihood.

However, most family firms are small in scale and produce a single type of product, which leads to the weak anti-risk capability and makes them vulnerable to dynamic situations. For instance, in the context of severe fluctuations in the global industrial chain and supply chain caused by the current global economic turmoil and the COVID-19 epidemic, many family firms, especially technology-based ones, have encountered serious challenges, such as the disruption of the supply of core raw materials and the disruption of the division of labor in the value chain. These firms are likely to be faced with the dilemma that normal production cannot be guaranteed and the market shrinks sharply. Therefore, the practical problem of how to deal with the impact of the turbulent situation and promote the better and faster development of the family firms is expected to be explored.

As a management tool for firms to effectively deal with risks and challenges, strategic entrepreneurship (SE) pursues the exploration of future business fields and the development of existing businesses at the same time (Webb et al., 2010), which means that it emphasizes the pursuit of new development opportunities through integration while pursuing current competitive advantages (Hitt et al., 2011). Therefore, it is considered to be an important approach for firms to capture opportunities (Withers et al., 2018), seek advantages and achieve sustainable development (Hitt et al., 2001).

The existing studies on SE in family firms have been discussed from the perspectives of resource orchestration (Chirico et al., 2011), inter-generational succession (Lee et al., 2019), family involvement (Bendig et al., 2020), internationalization strategy (Arregle et al., 2017; Zahra, 2020) and so on. Related studies have mainly focused on the relationship between family business control and SE (Boellis et al., 2016), the trans-generational entrepreneurial family firms (Nelson and Constantinidis, 2017; Clinton et al., 2018), the impact of SE on firm performance and strategy change (Arregle et al., 2017; Zahra, 2020), and the exploration and exploitation behavior in the family firms SE (Ireland and Webb, 2009; Hughes et al., 2021). There are few studies on the behavior mechanism of SE in family firms, and there is still a lack of understanding of why and how firms choose specific strategic entrepreneurial paths and behavior. This significant gap may make it difficult for existing theories to provide effective and clear action guidance for the SE of family businesses, which can lead to the practical problem that the managers do not know how to carry out SE activities.

In order to address this gap, this paper takes PX Electronics Co., LTD (hereinafter referred to as “PX Electronics”), a technology-based family business that has maintained good growth through strategic entrepreneurial activities in a dynamic context, as a sample case, and applies the grounded theory methodology to conduct an exploratory case study. PX Electronics has undergone two major strategic changes since its inception, and at each stage the entrepreneur was able to select appropriate strategic entrepreneurial paths and behaviors to effectively address various challenges. Therefore, we would like to discover the general rules behind this enterprise and provide reference for more family business strategic entrepreneurship. For achieving this objective, this paper aims to address the following research questions:

- Why do family firms entrepreneur choose this different strategic entrepreneurial behaviors and path at specific stages?
- How does entrepreneur’s social identity affect strategic entrepreneurship at various stages of business development?

Answering these questions is important for several reasons. First, it helps to clarify the common norms of the family firms strategy entrepreneurial path, and summarize the mechanism for such firms to achieve sustainable development. Second, it can also provide decision-making reference for entrepreneurs to exert their initiative, choose appropriate strategic entrepreneurial behaviors, and achieve rapid growth of family firms.

This article has the following research contributions. First, this study provides a new explanatory framework for the path selection mechanism of SE in family firms. Based on the social identity theory of entrepreneurs (Fauchart and Gruber, 2011; Powell and Baker, 2014; Wry and York, 2019), this paper constructs a strategic entrepreneurial path model for technology-based family businesses from the perspective of dynamic identity evolution. The mechanism of strategic entrepreneurial path selection and behavioral mechanism of technology-based family firms in different entrepreneurial contexts are explained, and provides a theoretical framework for future empirical research and theory development. Second, this study responds to the call for in-depth research on SL by scholars (Hallinger and Suriyankietkaew, 2018; Iqbal et al., 2018, 2020, 2021; Burawat, 2019), and expands the research related to SL behavior. This study finds that the SL of entrepreneurs plays an important role in the implementation of firms’ strategic entrepreneurial activities, and expands the application of SL in family firms entrepreneurial activities. Furthermore, this paper enriches the research on the entrepreneurial social identity literature. This study responds to scholars’ calls for research on the multiplicity and dynamics of entrepreneurial identity (Powell and Baker, 2014, 2017; Pan et al., 2019; Mmbaga et al., 2020), clarifies the dynamic evolution of entrepreneurial social identity with changes in entrepreneurial contexts, and explores the impact mechanisms of the evolution of entrepreneurial social identity on entrepreneurial behavior, which expands relevant research on entrepreneurial identity theory, and also provides a useful exploration of the subjective motivation of entrepreneurs in SE.

The remainder of this study is organized as follows. Section two reviews the literature on SL, SE and social identity of entrepreneur. Section three describes research methodology and research design. Section four is case analysis and data coding. Section five reports the case finding and research results. Finally, the article ends with conclusions and limitations, and at the same time presents directions for further research.

## Literature review

### Entrepreneur’s social identity

Entrepreneurial identity is a set of claims around the founders, organizations, and market opportunities of an entrepreneurial entity that gives meaning to questions of “who we are” and “what we do” (Navis and Glynn, 2011). In the research domain of entrepreneurial identity, role identity theory and social identity theory are two different theoretical perspectives concerned with self-concept and the nature of an individual’s normative behavior (Stets and Burke, 2000; Hogg et al., 2012; Zuzul and Tripsas, 2020). Social identity theory focuses on inter-group relations and explains how the behavior of individuals and groups is derived through self-categorization and social comparison processes (Tajfel and Turner, 1979; Hogg and Terry, 2000). Entrepreneurs’ long-term prominent identity type and identity structure determine the firms’ strategic response to adversity (Powell and Baker, 2014; Gruber and MacMillan, 2017), so this theory also explains how entrepreneurs take different behaviors in the face of similar environments (Fauchart and Gruber, 2011), and analyzes why entrepreneurs are more likely to connect with some groups than others (Powell and Baker, 2017).

Fauchart and Gruber (2011) divide the entrepreneur’s social identity into Darwinian, Communitarian and Missionary based on the social motivations, self-evaluation basis and individual frame of reference. The three social identity types encompass different levels of social inclusion, expanding from “self” economic interests to “our” community interests to “whole society” overall interests (Fauchart and Gruber, 2011; Sieger et al., 2016; Pan et al., 2019).

Entrepreneurs who fall into Darwinian category focus primarily on establishing strong and profitable firms, and their primary motive is to make profits and accumulate personal wealth. This makes them value a professional “business school” approach to creating and running a firm, and pay close attention to managing their firms according to solid business principles. They try to gain a competitive advantage by differentiating their firms from the competitors (Fauchart and Gruber, 2011; Powell and Baker, 2014, 2017; Mmbaga et al., 2020). Entrepreneurs with Communitarian-type social identity are enthused by their ability to contribute to the community with their innovative products and value the support they receive from community members during the entrepreneurial journey (Fauchart and Gruber, 2011; Gruber and MacMillan, 2017). Missionary founders believe that firms can be powerful agents of social change. Therefore, they are committed to being agents of social change, positively impacting the well-being of others, and acting in a responsible, transparent and empathetic manner (Fauchart and Gruber, 2011; Powell and Baker, 2014; Pan et al., 2019; Mmbaga et al., 2020).

When the social identity of entrepreneurs is consistent with the self-expectation, they will show more positive emotions (Murnieks et al., 2016) and entrepreneurial self-efficacy (Brändle et al., 2018). When the social identity of entrepreneurs is similar to the expectations of stakeholders, they can obtain more identification, trust and resource support from stakeholders (Busenitz et al., 2014; Porck et al., 2018; Ashforth Blake et al., 2020), and enhance the effectiveness of management (Ireland and Webb, 2007; Mmbaga et al., 2020).

### Identity and leadership

Akerlof and Kranton (2010) pointed out that individual actors use their power to control followers, and this old-model leadership is not only costly, but also has the signal of distrust, which can easily cause the division between each other (see also Akerlof, 2011). Recently, inspired by social identity theory (Tajfel and Turner, 1979) and self-classification theory (Turner et al., 1987), some scholars have proposed a social identity approach to leadership. It assumes that leadership is a social influence process that is structured by people’s social group memberships.

Leadership does not operate in a vacuum but centers on a sense of shared group membership between leaders and followers within a given social context (e.g., as members of a team, department, or organization). Here, the more leaders are attuned to the social identity that they share with followers (a sense of “we-ness”), the more influential and trusted they are likely to be (Barreto and Hogg, 2017; Van Dick et al., 2018). Many studies have supported these ideas and shown, for instance, that the more prototypical leaders are of the group that they are leading (i.e., the more they are seen to embody the norms, values, and goals of their group), the more effective they are securing more follower support, and having greater leeway to make decisions (Platow et al., 2015; Barreto and Hogg, 2017).

Based on this, some scholars put forward the construct of identity leadership (van Dick and Kerschreiter, 2016; Van Dick et al., 2018; Haslam et al., 2017). Because identity leadership is centered on power through followers (Turner, 2005), it is a more promising new leadership model. Employee perceived identity leadership is uniquely related to important indicators of leadership effectiveness, including employees relationship with their team (identification and perceived team support), well-being (job satisfaction and reduced burnout), and performance (citizenship and innovative behavior at work; Smith et al., 2018; Van Dick et al., 2018).

### Sustainable leadership

Sustainable leadership originated from Rhineland management (Avery and Bergsteiner, 2016) and effective leadership theory (Iqbal et al., 2018), in the assumption of which organizations are viewed as a part of an open system that emphasizes the responsibilities of the organizations to the society and stakeholders. As an emerging type of leadership, sustainable leadership contributes to the organizational performance in the context of current and future environmental, economic, and social goals(McCann and Holt, 2010; Iqbal and Piwowar-Sulej, 2022), sustainable leaders, stimulate and inspire followers focusing on their needs, and-like participative leaders-involve employees in decision-making. They use positive behaviors as a method to guide others which is in line with positive leadership(Salmi et al., 2014; Gerard et al., 2017; Iqbal and Piwowar-Sulej, 2022).

Sustainable leaders need to have a long-term perspective, corporate social responsibility and ethical behavior (Hallinger and Suriyankietkaew, 2018) to improve the lives of all company stakeholders and to generate current and future profits for the organization (McCann and Holt, 2010; McCann and Sweet, 2013). According to Ferdig (2007), the sustainable leaders act responsibly by comprehending and acting on sustainable issues irrespective of their formal leadership positions. Avery (2005) emphasized that sustainable leaders should promote systemic innovation in order to develop a skilled, engaged, and loyal workforce, deliver quality products and services, and add value. According to Slankis (2006), SL includes 10 pillars such as change orientation, high credibility, patience, translational skills, energy and passion, foster persuasiveness, mentoring, development.

As an effective leadership style to improve the competitive advantage and overall performance of an organization, sustainable leadership has impacts on many resources. It enhances knowledge sharing, development of employees, participation, and empowerment (Iqbal and Piwowar-Sulej, 2022; Iqbal and Ahmad, 2020; Gjerde and Ladegård, 2019). Finally, sustainable leaders construct positive narratives in organizational context leading to increase in subordinates’ energy (Di Fabio, 2017). This requires leaders to pay attention to the long-term well-being and stability of the organization in the decision-making process, so as to meet the needs of the current generation without compromising the needs of future generations (McCann and Holt, 2010).

Additionally, SL practices, including valuing employees, a shared vision, social responsibility, and friendly labor relations, can significantly drive long-term corporate performance (Suriyankietkaew and Avery, 2016). Sustainable leaders should focus on capacity building, sustainable change, and long-term outcomes, which allows them to look beyond immediate short-term interests to a larger context when pursuing sustainable development goals (Hallinger and Suriyankietkaew, 2018). SL enables organizations to learn better, faster, more flexible and more adaptable than their competitors (Hargreaves and Fink, 2012). However, SL is still in its infancy, and there is an urgent need to extend this domain in the literature (Burawat, 2019).

### Strategic entrepreneurship and family firm SE

Hitt et al. (2001) were first proposed the concept of strategic entrepreneurship, which has been in development for 20 years now. During this period, scholars have focused on the connotation, nature, resource management, and other aspects of strategic entrepreneurship have been and made great progress. Early research focused on a process perspective, which described strategic entrepreneurship as a successful combination of strategic management and entrepreneurship, including entrepreneurial actions taken from a strategic perspective and strategic behaviors taken from an entrepreneurial perspective, as well as creating more wealth for the firm (Hitt et al., 2001; Ireland et al., 2003).

Significant progress has been made in the following research. The concept of strategic entrepreneurship was subsequently enriched by different scholars in terms of elements and dimensions (Ireland et al., 2003; Hitt et al., 2011), entrepreneurial orientation (Dess and Lumpkin, 2005), and exploration and exploitation (Ireland and Webb, 2009). In particular, Ireland and Webb (2007) argued that SE is composed of two types of activities: entrepreneurial opportunity seeking (exploration) and strategic advantage seeking (exploitation). Schindehutte and Morris (2009) pointed out that strategic entrepreneurship is an independent paradigm and a conceptual domain of how decision-makers take advantage of the creative potential of complex dynamic systems. Simsek et al. (2017) emphasized that strategic entrepreneurship is a logical set of enterprise behavior decision-making system. Although scholars have given different descriptions of strategic entrepreneurship, leading to a blurring of the boundaries of strategic entrepreneurship, there is a basic consensus that strategic entrepreneurship is an organizational innovation that integrates opportunity-seeking and advantage-seeking behaviors (Ireland and Webb, 2007, 2009; Mazzeii et al., 2017).

Only by organically combining opportunity seeking and advantage seeking, and making a reasonable allocation of resources between the two type of activities, can the success of SE be achieved (Ireland and Webb, 2009; Mazzeii et al., 2017). The sustainable development of enterprises is not only a process of continuous opportunity seeking, but also a process of searching for strategic advantages through resource allocation. Therefore, the SE theory can provide a new perspective for the study of sustainable development of enterprises by organically integrating the value creation behavior and advantage construction behavior of enterprises.

In the strategic entrepreneurship theory, through the integrated research on entrepreneurial behavior and strategic behavior, on the one hand, it can use entrepreneurial behavior to identify and develop entrepreneurial opportunities, enabling enterprises to enter new markets or develop new products and services to seek greater value creation. On the other hand, through strategic behaviors, it can help explore the key resources and resource allocation for enterprises to build competitive advantages in an uncertain dynamic environment, so as to achieve the organic integration of corporate value creation and competitive advantage construction (Hitt et al., 2001; Luke and Verreynne, 2006).

Research on SE in family firms has received more academic attention after 2011, the related studies focus on resource orchestration and strategic entrepreneurial performance in family firms (Chirico et al., 2011), inter-generational succession and SE (Nelson and Constantinidis, 2017), family involvement and entrepreneurial decision (Boellis et al., 2016; Arregle et al., 2017), and other aspects. However, the previous literature has not thoroughly explored the path selection and behavioral mechanisms of family firms in special stages of SE. This may make it difficult for the existing theories to provide effective and clear action guidance for the SE of family firms, and the company does not know how to promote its SE at different stages and to take full use of the dual advantages of strategy and entrepreneurship. Therefore, the purpose of this paper is to explore how and why family firms choose different strategic entrepreneurial paths in dynamic contexts, so as to effectively address risk challenges and contribute to sustainable business growth.

### Research review

The literature review found that the content and objects of the research on SE of family firms are diverse and cross-disciplinary. Researchers have conducted studies from multiple perspectives to strengthen the micro-foundations of entrepreneurship theory. They analyzed the motivations and outcomes of SE, but there is a lack of research on the paths of SE. Although scholars recognize that entrepreneurial identity has an important impact on entrepreneurial behavior and corporate strategy, and that appropriate identity narratives can enhance entrepreneurial leadership, managerial effectiveness, and resource integration capabilities. However, there is few researches on the diversity and dynamics of identities, especially how entrepreneurs develop and dynamically evolve their identities (Leitch and Harrison, 2016), and the impact of identity dynamics on leadership remains to be studied in depth.

## Materials and methods

### Method and case selection

#### Method selection

The longitudinal single case study research was chosen in this paper for the following reasons.

First, the purpose of this study is to answer the questions of how family firms achieve sustainable growth in highly dynamic market environment, and how and why entrepreneurs can choose various paths for SE at a specific stage in the development of the enterprise. A dynamic process and a longitudinal single case study can help to understand the dynamic evolutionary process (Pettigrew, 1990; Yin, 2014). Second, the questions of this study include “why” and “how” category, and the previous literature does not adequately answer such questions, so case studies are suitable for answering this question (Yin, 2014). Third, this paper adopts the theoretical construction paradigm of putting forward the relevant propositions by means of the case analysis, and the case study research is a suitable method for this paradigm (Eisenhardt and Graebner, 2007; Eisenhardt, 1989). Fourth, in terms of the number of cases, it is appropriate to adopt the longitudinal analysis of a single case because of the need to analyze the relationship between the evolution of different specific entrepreneurs’ social identity, sustainable leadership and strategic entrepreneurial behavior. This can more clearly demonstrate the evolution mechanism between various constructs.

#### Case selection

In order to construct a theory, the case selection is usually made adopting theoretical sampling rather than statistical sampling, and the cases need to be representative and heuristic. After many in-depth discussions and arguments, PX Electronics, which is engaged in the R&D and production of nanocrystalline soft magnetic materials in the magnetic material industry, was chosen as the case of this study.

This is due to the following reasons: Firstly, PX Electronics has effectively met the risks and challenges and achieved rapid expansion through SE. Since its establishment in 2008, it has effectively dealt with the challenges of various risks and achieved profitability by using its technological advantages. In 2016, the company has achieved expansionary growth, which is highly typical and inspiring. Secondly, PX Electronics is a technology-based start-up family firm, where entrepreneur participate in the creation, growth and expansion of the company throughout the process. It is suitable to analyze the strategic entrepreneurial process of the company from the perspective of the evolution of the entrepreneurs’ social identity. Thirdly, the magnetic material industry is technology-intensive with strong linkages to the upstream and downstream firms of the value chain. The competition among enterprises around technological advantages is fierce, which makes it an ideal industry for strategic entrepreneurial research in technology-based family businesses. Fourthly, the research team of this study has been tracking and paying attention to the development of PX Electronics for a long time, and has provided long-term management consulting services for the company, which can also ensure the availability and reliability of the research data in the study.

### Case company

#### PX electronics

Founded in June 2008, PX Electronics is located in Fengcheng Industrial Park, Shanghai, and it is a high-tech-based family firm integrating R&D, production and sales of nanocrystalline soft magnetic materials. The main products include amorphous, ultra-microcrystalline magnetic cores, cobalt-based amorphous magnetic cores and so on, which are widely used in the information communication and power electronics industries and have gradually become the core materials for high-end manufacturing products such as aerospace, new energy, electronic power, and medical care. These products have been used in the production of sensors of high-frequency transformers, inverters, inductors, electronic components, various magnetic components in power control systems, and magnetic components for telecommunication equipment and pulse power devices. The core raw material is ultra-fine crystal strip. In 2016, the company achieved scale expansion and established CL Electronics Co., Ltd. (hereinafter referred to as “CL Electronics”) in Shandong Province, mainly focusing on the R&D and production of ultra-microcrystalline strips.

#### The staged characteristics of case company

According to the entrepreneurial process of PX Electronics, combined with the theory of multi-stage entrepreneurial process, the entrepreneurial process of PX Electronics is divided into four stages.

##### The entrepreneurial planning stage (2006–2008)

After graduating from university in 2001, the entrepreneur joined Beijing Q Company (a technology-based company engaged in the R&D and production of electronic components) and has been engaged in technology research and development and technical services for nearly 7 years. This work experience enables the entrepreneur to master the core technology of nanocrystalline soft magnetic material design, research and development, has strong technical advantages, and lays a solid foundation for subsequent entrepreneurship. In 2008, the entrepreneur resigned from Beijing Q Company and came to start his own business in Shanghai.

##### The initial stage (2008–2011)

At this stage, the company experienced a series of fundamental activities including enterprise creation, market development, and product R&D. By strengthening the management of customers, suppliers and partners, the company actively builds product reputation and obtains market legitimacy.

##### The entrepreneurial growth stage (2011–2015)

After the practice and operation in the start-up period, the business and orders of company was increased, but the supply of raw materials and production capacity faced serious challenges. At this stage, the company has improved its profitability and performance through a series of changes such as activity optimization, quality control and value chain disintegration.

##### The expansion stage (from 2016 to date)

In order to cope with the delay in order delivery and decline in product performance caused by the untimely supply of raw materials and unstable quality in the procurement process, the entrepreneurs made a strategy of value chain vertical integration in 2016 after a comprehensive study and judgment. CL Electronics was then established to focus on the R&D and production of ultra-microcrystalline strips, which effectively alleviated the quality problems faced by PX Electronics in the procurement of raw materials. Since 2020, the company has added 3 production lines to effectively meet the growing market demand, and the products have been continuously recognized by customers.

### Data collection and processing

#### Data collection

Throughout the study, the researchers maintained a cautiously supportive neutral tone to minimize respondents’ social expectation bias. Following grounded theory protocol, a core initial interview guideline is applied to guide the semi-structured interviews. An interview guide merely helps interviewers keep conversations within the realm of the study, and it allows interviewers to adapt to where participants wants to tell their stories. Data collection process for the nanocrystalline soft magnetic industry and PX Electronics spanned nearly 2 years. In order to improve the reliability and validity of the case study, this study applies the triangulation method to analyze the PX Electronics case from multiple sources of information to ensure the reliability of the data (Yin, 2014). It includes formal in-depth interviews with the entrepreneur of PX Electronics and some senior managers, additional informal meetings and conversation, field observations, and hundreds of documents, images and artifacts.

##### Interviews

Interviews all began by making introductions, explaining the basic research purpose without revealing any preconceived notions or working hypotheses, outlining the administrative details about data collection, analysis, storage, confidentiality, and obtaining informed consent. Formal interviews lasted 1 to 2 h, during which the research team conducted semi-structured interviews with entrepreneur, family members, senior managers and employees. Interviewers asked to hear about any difficulties the founders faced in their day-to-day activities and about how they addressed those difficulties. The questions cover the entrepreneur’s mental journey, the development stage of the company, technology R&D, raw material supply, product production and sales. As part of telling the firm’s stories, the founder provided extensive biographical data that stretched long before the target business was founded. All interviews were recorded and transcribed, the supplementary interviews were conducted for any ambiguities and discrepancies. All interviews were professionally transcribed, and the average interview length was 85 min, with a range of 48 min to 5 h.

##### On-site observations and conversation

The researchers conducted on-site visit as supplemental data, including facilities tours and plant visits, which allowed the researchers to engage in unobtrusive observation of interactions between employees and various stakeholders, as well as with the founder. Moving into the topics of conversation, participants were asked to describe their roles and backgrounds followed by their views on what their organization stood for. During the process, researchers explored more details and stories around what seemed important to participants.

##### The documents

Analyzed data also includes those from secondary data sources such as trade publications, websites, annual reports, brochures, patent filings, company archives, financial statements, historical video footage and social media activity, displays of historic label and other internal documents. In addition to collecting marketing and business documents, hundreds of photographs and copious field notes were taken. The details of data collection are shown in Table 1.

**Table 1:** Summary of data collection.

Date	Days	Data source	Content
2018/10	3	Company website, media public information, industry forums	Get a preliminary understanding of the case companies and develop a research framework
2018/10	0.5	Open-ended interviews with entrepreneurs	Negotiate a detailed interview plan and specific arrangements
2018/11	2	Onsite observation; in-depth interview; archival material	In-depth company site visit, understand the company’s development history, listen to family members’ comments on entrepreneurs (3 h); experience the product production process (1 h); in-depth communication with grass-roots employees to understand their specific job responsibilities, work content, etc. (2 h)
2018/11	2	Publicity material; meeting records	Conducting filed survey of production lines and warehouses (4 h); interviews with company executives and relevant vice presidents (6 h); look through company files (4 h).
2019/02	1	Workshop visits; field survey; staff interviews	The team members visited the front line of the workshop to learn about the technological process and production operation, and communicated with the employees to learn about their welfare benefits and the evaluation of the entrepreneurs, etc.
2019/06	1	Feedback Communication; in-depth interview	The team members work in two groups. The first group continues to conduct in-depth interviews to supplement and improve the information; the second group provides feedback to the enterprise for all the data compiled in the preliminary coding to improve the accuracy of the information.
27/2019/12	0.5	Informal interview with entrepreneur	Communicate with entrepreneurs in an informal setting to learn about recent developments in the company.

#### Data processing

In accordance with the method and process of the exploratory case (Eisenhardt and Graebner, 2007), the data processing is carried out as follows. Firstly, after each interview, the interview data was transcribed as quickly as possible, the unclear or uncertain problems were identified, and the key points for the next interview were listed. Secondly, Interviewers also gathered secondary data to describe contingencies (industry, tax structure, or environment) and for triangulation purposes (i.e., corroborate information gathered through interviews). Examples include web sites, annual reports, press articles, and available internal documents. This enabled the teams to get a more comprehensive picture of the families, the firms, and their activities as a whole. Thirdly, according to Yin (2014), it adopted the analysis strategy of the identity and behavior matching of entrepreneurs under different time nodes, to study the sustainable development model and innovation mechanism of PX electronics company; Fourthly, following the principles of problem orientation, triangulation verification and avoidance of subjective preferences, the research team members extracted the research results through repeated discussions and screening on the premise of no prior assumptions or theoretical viewpoints and on the basis of ensuring that the logical relationship is supported by at least two or more sets of data.

## Case analysis

### Coding

Based on grounded theory (Strauss and Corbin, 1998; Corbin and Strauss, 2015), data coding followed the principles of theoretical sampling and was carried out through three steps: open coding, axis coding and selective coding. By doing so, it can explore emergent themes, collect additional data, and maximize observational opportunities.

#### Open coding

Open coding is a process of analyzing data to extract thematic categories and their characteristics. First, it disintegrates and organizes the original data and discourses obtained by the investigation according to the sequence of events, to discover and refine relevant constructs in the events, and assign construct labels. Second, related constructs were clustered into first-order concepts. According to the stage of the firm development, we extract the events related to the research topic of this paper from the original data to form relevant constructs, and retains the constructs which appear for three times or more to determine the first-order concepts. After sorting and analysis, 67 constructs and 42 first-order concepts were extracted. Table 2 shows partly first-order concepts formed through open coding.

**Table 2:** Example of some first-order concepts generated by open coding.

Stages	First-order concepts	Constructs	Coding examples
Initial stage	creation of for-profit ventures	Entrepreneurship; profit	*“I was trying to use my skills to start a business, improve the economic situation and provide a good life for my family.”(Interview with entrepreneur)*
	Innovative cooperation model	Flexible; customized manufacturing	*“I agree that the payment for goods can be paid one cycle later. I bought raw materials with his deposit, and conduct R&D and production according to the requirements, and then got the second batch of orders after passing the inspection… Orders are gradually increasing.”(Interview with entrepreneur)*
	Labor cost advantage	Social relations; high coordination efficiency	*“*…*they (family members) all work in the company, which can reduce some labor costs and facilitate management*…*”(Interview with entrepreneur)*
Growth stage	Complementary advantages	Outsourcing; cooperation	“*We outsource some orders that we are not good at to our peers, and they also introduce us to some orders that we are not good at.” (Interview with entrepreneur’s wife)*
	Open suggestions	Accept suggestions; smooth communication	There were a lot of suggestions from employees about the wide variety of order types at the time. (meeting records)
	Performance improvement experiments	Active cooperation; data collection	*“Han (workshop manager) and others also helped me collect data and put forward suggestions for improvement. We improved the technical requirements of key links, and product performance and competitiveness were greatly improved.” (Interview with entrepreneur)*
Expansion stage	Respond to community concerns	Peer encouragement; community demand	“*Many peers are facing the same dilemma of unstable raw material quality and cannot find an effective solution. Once, a peer asked me, if you have a technical advantage, why do not you try to produce your own strips? “(Interview with entrepreneur)*
	Environmental consciousness	Recyclable; waste discharge	*“In production, we pay great attention to the safe discharge of waste gas and waste water, and use recyclable packaging boxes when transporting products.”(Interview with entrepreneur)*
	Cost allocation	Channel sharing; technology sharing	*“*…*the two companies can share resources in terms of technology, sales, advertising and marketing, and allocate costs. (Interview with entrepreneur)*

#### Axis coding

The task of this stage is to refine the internal connections between multiple first-order concepts. In line with the logic paradigm of “condition-behavior-result,” multiple first-order concepts are correlated with find logical relationships between them, and the correlated themes are classified into the same second-order theme. In-depth analysis is performed on one category at a time to discover the relationships between first-order concepts and second-order themes. The same approach is used to discover and establish associations between second-order themes and aggregate dimensions. For example, the constructs such as “management cost control and labor cost control” are conceptualized into the first-order concepts of “cost advantage,” and the first-order concepts of “cost advantage” and “efficiency advantage” are then categorized into the second-order themes of “advantage seeking,” after which the “advantage seeking” and “opportunity seeking” are integrated into the aggregated dimension of “SE” to form a complete chain of evidence, as shown in Table 3.

**Table 3:** Example of partly aggregate dimension generated after axis coding.

First-order concepts	Second-order themes	Aggregate dimensions
Creation of for-profit ventures Pursue private economic goals	Darwinian identity	Entrepreneur’s social identity
Complementary advantages Information Sharing	Communitarian identity	
Balancing long-term and short-term goals Change orientation	Systems thinking	Sustainable leadership
Innovation awareness Continuous learning	Open innovation	
New customer acquisition New product development	Opportunity seeking	Strategic entrepreneurship
Cost advantage Efficiency advantage	Advantage seeking	

After the constant comparison and induction, the 42 first-order concepts obtained from open coding were integrated into 27 second-order themes and then merged into three aggregate dimensions, they are entrepreneur’s social identity, SL and SE. The connotation and nature of the three aggregation dimensions are described as follows.

##### Entrepreneur’s social identity

The construct of entrepreneur’s social identity is named with reference to the views of Fauchart and Gruber (2011). Entrepreneur’s social identity may help explain why entrepreneurs facing similar contexts may act differently through self-categorization and social comparison. In this case, the social identity of the entrepreneur presents a “Darwinian” identity at the initial stage, a “Communitarian” identity in entrepreneurial growth stage, and a “Missionary” identity in the expansion stage.

##### Sustainable leadership

The construct of sustainable leadership is named with reference to the views of Iqbal et al. (2020). Sustainable leadership is a summary of series of effective leadership approaches for entrepreneurs in the qualitative materials to keep an open mind in the entrepreneurial process, take the interests of all stakeholders into consideration, balance short-term and long-term goals, and enhance the competitive advantage and overall performance of the organization through appropriate resource arrangement.

##### Strategic entrepreneurship

The strategic entrepreneurship is named with reference to the views of Ireland and Webb (2007). Strategic entrepreneurship is a summary of a series of activities in qualitative materials that entrepreneurs seek to upgrade their technological advantages and seek for entrepreneurial opportunities through resource integration, value chain management, process optimization and other activities based on different entrepreneurial situations.

#### Selective coding

In the selective coding step, it aims to analyze the relationship between aggregate dimensions, refines core categories, and builds grounded theoretical models. The key to this process is to explore and discover a “story line” that can play the role of “outlining” from the aggregate dimension and string all categories into a core category. By constant comparison of the obtained aggregate dimensions with existing theories, it is found that the core category of this paper can be expressed as: the evolution of entrepreneur’s social identity affects strategic entrepreneurial behavior in a specific period through sustainable leadership. The “story line” around this core category can be summarized as “entrepreneur’s social identity—sustainable leadership—Strategic Entrepreneurship.” The theoretical model of this paper is shown in Figure 1.

**Figure 1:** Theoretical mode.

### Saturation test

This study takes more than 1 year to collect the data. To further enhance trustworthiness of the data, triangulation method was used to cross-validate the qualitative data collected from different information sources. During the process, the data was continuously supplemented, checked and verified, and supplementary communication with the company’s entrepreneurs has been carried out in a timely manner on certain issues for many times. After the completion of data processing, it took about 6 months to conduct a return visit to the enterprise and obtain the review feedback of family firms members on these reports. According to the feedback, appropriate adjustments and improvements have been made to the relevant data. Finally, in order to ensure the theoretical saturation, another third of the reserved interview records were used to test, and no new categories and relationships were found. Therefore, it can be considered that the core categories and theoretical models of this case have reached saturation.

## Finding

The serious challenge for today’s organizational leaders is to successfully guide their organizations through volatile economic times and deal with the topic of sustainability (Fable et al., 2005). If the organization is perceived as a living system, it is expected to continually evolve and adapt over time. The goal of traditional leadership’s goal was to stay on course. However, maintaining the same strategy during times of change can be disastrous. Exceptional corporate leadership must therefore remain in a flexible, fluid state to encourage and nurture creativity and innovation (McCann and Holt, 2010).

From the qualitative materials of PX Electronics, it can be found that during the entire entrepreneurial process, entrepreneurs flexibly and dynamically adjust their social identity according to changes in the internal and external situations of the enterprise, so as to improve their sustainable leadership, and promote the implementation of enterprise strategic entrepreneurial behaviors and activities to ensure the sustainable growth of the enterprise.

In the entrepreneurial planning stage, based on prior experience and self-assessment, entrepreneurs identified entrepreneurial opportunities, actively construct an entrepreneurial identity, completed the transition from employee identity to entrepreneurial identity, and laid the foundation for entrepreneurial activities.

In the start-up stage, benefited from Darwinian social identity and his technical advantages, entrepreneur was driven by vision, actively persuaded stakeholders to obtain necessary resource support, and quickly transform their technological advantages into products through SL behaviors such as team building and resource deployment to obtain economic benefits.

In the growth stage, based on Communitarian identity, the entrepreneur, through systematic thinking, considered both long-term and short-term interests, cooperated with community members, and divided the value chain horizontally, as well as focused on product performance improvement. Besides, the entrepreneur optimized management process, and carried out opportunity search and advantage search activities for SE.

During the expansion stage, entrepreneur responded to community concerns, and through vertical integration of the value chain, transferred the technological advantages to upstream raw material production based on the Missionary social identity. In addition, entrepreneur also integrated downstream products and carried out strategic entrepreneurial activities. In this case, the entrepreneur’s social identity evolves with the development of the enterprise, and this evolution prompted him to adopt different SL methods according to the changing situation as well as promoted the implementation of strategic entrepreneurial behavior, and finally led to the achievement of the goal of sustainable development of the enterprise.

### Entrepreneurial identity construction (the entrepreneurial planning stage: 2006–2008)

During the entrepreneurial planning stage, based on previous experience and self-assessment, entrepreneurs identified entrepreneurial opportunities, completed identity transformation, and constructed entrepreneurial identity through identity prototype reference and industry insights.

Entrepreneurship enables entrepreneurs to freely pursue their dreams and goals in the process of business creation (Fauchart and Gruber, 2011), realize personal value by aligning “who I want to be” with “what I can do,” so entrepreneurial behaviors are, to a significant extent, the expression of one’s identity (Gruber and MacMillan, 2017). In the entrepreneurial planning stage, active and conscious identity construction enables entrepreneurs to quickly complete identity transformation and realize the synergistic effects of personal entrepreneurial efforts, self-identity and external support. The active construction of the entrepreneur’s identity is the basis for the formation of the entrepreneur’s identity and the development of entrepreneurial activities (Navis and Glynn, 2011).

Long-term experience accumulation and continuous learning enable entrepreneurs to have keen industry insight and opportunity perception. The case data code shows that in the entrepreneurial planning stage, the entrepreneur has been engaged in technology R&D and technical services for 7 years in Beijing Q Company. 7 years of work accumulation not only enabled the entrepreneur to master the core technology of nanocrystalline soft magnetism, but also established a close personal relationship with his mentor. Through the experience and self-assessment, the entrepreneur perceived the entrepreneurial opportunity when the Chinese government introduced a number of supportive policies and preferential measures in credit, taxation, land leasing and administrative approval. As a result, the entrepreneur resigned from Beijing Q Company and chose to build a factory in Fengxian District, Shanghai, which has a strong entrepreneurial atmosphere and a good business environment, completing the transition from a technical employee to an entrepreneur.

### Entrepreneur’s Darwinian identity, SL and SE (the initial stage: 2008–2011)

#### Entrepreneur’s Darwinian identity and SL

In the initial stage, the main motivation of entrepreneurs is to build a profitable enterprise, to accumulate personal wealth, to meet personal economic goals and ultimately to maximize income, so as to create a better living environment for their families. Therefore, entrepreneurs in this period mainly presented a Darwinian social identity. However, like other start-ups, PX Electronics also faced issues such as lack of resources, legitimacy and market. The entrepreneur recognized the need to obtain the necessary resource support through social relationships if the creation of the business was to be accomplished quickly. As a result, the entrepreneur changed his orientation, obtained resource support from his families through active persuasion behaviors, and tried a series of innovative cooperation models and skills transformation behaviors to improve adaptability and carried out effective entrepreneurial behaviors to overcome difficulties.

First, vision-driven. Based on a shared vision, entrepreneur provided a business plan and roadmap to convince family members to let them understand the feasibility of the business plans, and obtained emotional encouragement and resource support from family members. At the same time, based on shared interests, entrepreneur promised fixed and guaranteed income to attract like-minded employees to join the company and build entrepreneurial team. Secondly, based on shared interests and open innovative awareness, entrepreneur innovated cooperation models, gained the trust of potential stakeholders, obtained the necessary resource support, accelerated the development and production of initial products to obtain market legitimacy. The creation of a profitable business was accomplished through this series of SL action. The references to relevant representative materials are shown in Table 4.

**Table 4:** Typical examples and coding results for the initial stage (partial).

First-order concepts and typical examples cited	Second-order themes	Aggregate dimension
Creation of for-profit ventures *“I just want to use my technological advantages and social relations to start a business while I’m young. If I succeed, my family can also have a good life.” (entrepreneur)”* Pursue private economic goals *“My purpose at that time was to make money, build my own financial wealth, and achieve the purpose of personal wealth accumulation”(entrepreneur)*	Darwinian identity	Entrepreneur’s social identity
Produce competitive products *“I look forward to the opportunity to use the technical advantages accumulated from previous work to produce competitive products and gain more markets and customers. (entrepreneur)* Self-evaluation and competition with other firms “*Using my working relationships, I also learned about some products from other companies in the same industry and compared the products I tested with theirs, and found that the quality was similar, which gave me a lot of confidence.” (entrepreneur)*		
Prepare a business plan “…*According to national policies and my industry knowledge, I made a clear business plan. When I told them (family and friends) about my plan, they also felt good after listening to it”(entrepreneur)* Team building (persuading and hiring employees) *“I was doing technical work on TV filters in another company at the time. Later, my brother started a business. I knew that he was very skillful in terms of technology. Now the salary is much better than before” (the younger brother of the entrepreneur’s wife)* Stable and substantial income *“He (entrepreneur) told me that the logistics industry is not easy to do. If I come to the company, I can have a stable job, the salary promise to me is also good, and I can have more time to take care of my family” (Interview with manager Han)*	Vision-driven	Sustainable leadership
Innovative cooperation mode *“I agree to pay for the goods with a one-cycle lag. I used the deposit to buy raw materials, and conduct R&D and production according to the requirements. After passing the inspection, I got the second batch of orders… We ship the goods every two or three days, so they do not worry about us. After a long time, this customer was fixed.” (entrepreneur)* Resources deployed *“In the initial stage, the company has limited capital and no money for automatic equipment, and many processes needed to be done manually. We invested most of our money in heat treatment and magnetization links, and some self-made and improved tools and equipment were used in other links” (entrepreneur)*	Innovation awareness	
New customer acquisition *“After the product was put into use, the customer feedback was good, and gradually it gained a certain market reputation, and developed several new customers” (entrepreneur)* New product R&D *“During product development, my wife’s brother, and manager Han have been involved in the testing of samples, and customers have also provided us with feedback, and the product has been finalized soon” (entrepreneur)*	Opportunity seeking	Strategic entrepreneurship
Cost advantage *“When the company was established, they (family members) all worked in the company to hope to provide some help, which saved a lot of labor costs; family members and Manager Han followed me for a long time, and the core workforce was relatively stable, saving a lot of recruitment and training costs.” (entrepreneur)* Dynamic and quick response capability *“If there is a new product production demand, it is only necessary to adjust the key links of the original production line and provide corresponding technical training to the employees.” (entrepreneur)*	Advantage seeking	

#### SL and SE in initial stage

Opportunity seeking and advantage seeking are two dimensions of SE (Ireland et al., 2003). In the initial stage, the SL has positive effects on opportunity seeking and advantage seeking.

Opportunity seeking refers to the opportunity discovery and creation activities of entrepreneurs based on technological advantages, through a series of technology embedding, process improvement, new product development, product performance improvement and new market development through product performance analysis, testing, R&D, etc. (Ireland and Webb, 2007). At this stage, opportunity seeking is mainly reflected in the entrepreneurs’ own technological advantages and the premise of common interests, integrating internal and external resources to complete the creation of new enterprises, acquisition of new customers, and research and development of new products.

The entrepreneur used the identity narratives appropriately to convince family members and potential stakeholders of their optimistic expectations and resource support. In the development of the first order, the entrepreneur used the influence of his original role at Beijing Q Company to gain the initial trust of the client. In order to eliminate the client’s doubts and win the cooperation opportunity, the entrepreneur innovated the cooperation model and agreed that the other party would first give him a small portion of the funds to buy raw materials. Then the client decided whether to continue the cooperation based on the performance after the samples were sent for inspection, and finally got the first order. After the funds were in place, raw materials were purchased in a short time to start research and development, and manager Han and the brother of entrepreneur’s wife then actively cooperate with the experiment to help the entrepreneur to quickly produce samples. After the trial, the entrepreneur made improvements based on customer feedback and suggestions, shortened the product development cycle, quickly passed the customer’s quality inspection, gradually established the market legitimacy, and received more orders.

Advantage seeking is the process of strategic management of resources that can generate sustainable competitive advantage (Ireland et al., 2003), including the stages of assembling, attracting, combining and transforming of resources (Brush et al., 2001). At this stage, the search for competitive advantage is mainly reflected in the fact that the entrepreneur attracted, assembled and combined the social resources required for entrepreneurship based on social relations and their own technological advantages, so as to achieve the purpose of reducing costs and increasing efficiency and gain market competitiveness.

Sustainable leadership enhances the dynamic capabilities of enterprises, enabling them to rapidly allocate and integrate resources to gain a competitive advantage. In the initial stage, family members and relatives working in the company were conducive to improving team stability, reducing management costs, and improving management decision-making. From factory site selection to equipment purchase, the entrepreneur strove to persuade factory owners and equipment suppliers to seek innovative cooperation models based on long-term shared interests, which relieved the cost pressure in the initial stage of entrepreneurship. The factory building was leased under the guarantee of a friend, and it was agreed that the rent would be paid after half a year; the equipment was obtained from a supplier who was acquainted with from the previous job by paying a part of the deposit first, and the balance was paid in batches later. In order to cope with the financial constraints, the entrepreneur mainly used limited resources to allocate the equipment related to the production line of heat treatment and magnetization, which can highlight the technical advantages, while other segments mainly meet the demand by improving some simple equipment. This resource integration strategy enables the enterprise to have a certain rapid response capability and flexible production capacity in the early stage of the business, which reduces the fixed investment risk. During the research in the workshop, some dusty equipment was found in the corner of the warehouse. Manager Han said that equipment like these were used at that time, and if there were new types of products to be produced, it was only necessary to adjust the key aspects of the original production line and train the staff accordingly, without purchasing some new tools, which could minimize the cost at that time.

This study also confirmed the existing research conclusion and further deepens the findings. It has been found in previous research that sustainable leadership practices, such as a strong and shared vision, were significant drivers and positive predictors of enhanced long-term firm performance (Suriyankietkaew and Avery, 2016), and this finding is also confirmed in this study. This study also finds that sustainable leadership practices can effectively promote the implementation of strategic entrepreneurial behavior, and ultimately improve overall enterprise performance (Sahai and Mahapatra, 2020; Iqbal and Piwowar-Sulej, 2022) through the opportunity-seeking and advantage-seeking activities of the enterprise such as new customer acquisition, new product R&D, cost control and quick response capability.

The references to relevant representative materials are shown in Table 4. Therefore, this paper proposes:

**Proposition 1:** In the initial stage, based on the Darwinian social identity, entrepreneurs can search for entrepreneurial opportunities and competitive advantages through sustainable leadership methods, such as vision-driven and innovative thinking to achieving resource acquisition, and promote the implementation of SE.

### Entrepreneur communitarian identity, SL and SE (the growth stage: 2011–2015)

In the growth phase, the interdependence between companies and community members increases, and many technical and market issues need to be solved by joint collaboration. Therefore, the social identity of entrepreneurs gradually changes to a Communitarian identity. This means that new and more valuable products and services are likely to be developed to enhance the competitiveness of enterprises and to achieve sustainable development through the division of labor, complementary advantages and information sharing with community members.

#### Entrepreneur communitarian identity and SL

After 2011, enterprise production management faced new challenges with the significant increase in business volume. For example, problems such as the wide variety of products and the untimely supply of raw materials have affected the continuity of production and the stability of product performance. Product variety also prevents businesses from achieving economies of scale, thus increasing equipment and overhead costs and reducing workers productivity. In addition, it also increases distribution costs, as the firm has to deliver each type of product in smaller batches and also need to maintain a certain amount of additional inventory to deal with unexpected changes in consumer demand across varieties. Furthermore, Shanghai’s strict environmental supervision and production restrictions for major events have brought challenges to the continuous production and on-time delivery, so the company often need to work off-peak and overtime, which led to many complaints from employees and frustrated work enthusiasm.

Therefore, the entrepreneur changed the mindset and seek to improve the status quo. First, cooperative innovation and continuous improvement. Entrepreneur actively learned the advanced experience of peers, and improved efficiency through process optimization. He then sought to improve product performance through knowledge absorption and innovative experiments. At the same time, he actively sought the help of community members by using his Communitarian identity, and sought peer OEM for some orders that cannot be completed on time, so as to maintain a normal supply order. Second, Valuing employees. The entrepreneur advocated employee participation in management to enhance their involvement and efficiency, and also built an atmosphere of trust for an open voice within the organization. This amicable labor relations encouraged employees to think and speak critically and differently, and in which the entrepreneur could receive constructive and feasible input.

In the archives, it can be found in a meeting record that everyone in the meeting expressed their opinions on the problems of complicated orders, serious overtime, and chaotic product accumulation.

“*In the past, we took some orders only because there was no other choice when the company was just established. Now that there are more orders, we should choose those orders that we are better at.”(Manager Han)*

“that there were too many product models, and tools and raw materials needed to be changed frequently during production, which seriously affected production efficiency, and sometimes it was easy to mix materials.” (a workshop worker)

“…with too many types, it was more difficult to find and deliver goods, and it was easy to send the wrong goods, which brought many unexpected problems.”(warehouse manager)

After systematic thinking and consultation with family members, the entrepreneur decided to adopt the suggestions of the employees, and made the decision to disintegrate the value chain horizontally to achieve a balance between short-term and long-term goals. Horizontal disintegration of the value chain refers to the value management model in which non-core activities in the value chain are transferred to other firms through licensing, outsourcing or transfer (Acemoglu et al., 2010). Through the division of labor and collaboration with community members, non-core businesses, such as logistics, accounting, advertising, certification, etc., were outsourced, and some low-profit or small orders were sought out OEM by peers. In this way, core resources can be concentrated in the links that exert technical advantages.

Communitarian identity empowers the entrepreneur’s SL and resource allocation capabilities during this period. On the one hand, Communitarian identity helps the entrepreneur gain the trust and support of external stakeholders; On the other hand, long-term cooperation promotes the complementarity and division of labor among community members. The entrepreneur always gets along with integrity and treats community members with courtesy and fairness, so they can maintain a good community relationship. Therefore, in the process of horizontal disintegration of the value chain, peers are willing to accept orders transferred by the entrepreneur, and will also transfer or introduce some orders that the entrepreneur is good at. Meanwhile, the entrepreneur’s integrity and compliance make suppliers willing to give priority to ensuring the company’s needs for raw materials, accessories and after-sales service.

#### Sustainable leadership and strategic entrepreneurship in growth stage

In the growth stage, based on the Communitarian identity of the entrepreneur and the status quo of enterprise development, the entrepreneur made an important strategic decision of value chain horizontal disintegration through a series of SL behaviors such as systematic thinking, innovation and continuous improvement, which promoted the implementation of enterprise SE. In this part, this paper will discuss the impact of value chain horizontal disintegration, a SL behavior, on the opportunity seeking and advantage seeking of SE.

Value chain horizontal disintegration has a positive impact on the enterprise’s opportunity seeking. First of all, after the value chain horizontal disintegration, entrepreneur can condense their core business, focus on product improvement trials in advantageous links, improve product performance and production capacity, and provide more possibilities for new R&D development and new order acquisition through reputation transfer.

*“In the past, for example, due to the variety of product models, the process essentials of each type of product could not be effectively controlled in the high-temperature crystallization process, resulting in unstable overall performance.”(entrepreneur)*

After the disintegrate of the value chain, the entrepreneur carried out iterative experiments in the core technology links, which enabled him to gradually produce products that met the technical requirements of the placement density, auxiliary material ratio and dynamic temperature control of different types of products in the heating furnace.

*“a regular customer increased the share of orders placed with us from 30% to 70%, and two key customers handed over some new orders to us for research and development, the total volume of orders does not drop but rises after the value chain horizontal disintegration.”(entrepreneur’s wife)*

Secondly, the horizontal disintegration of the value chain enhances the division of labor and knowledge flow among community members, and improves the availability of market information and advanced technologies for entrepreneur. The entrepreneur embedded some new technologies into the experiments of product performance improvement, which promoted the application of technological advantages, and ultimately met new customer needs to obtain more profit streams. The relevant representative citations are shown in Table 5.

**Table 5:** Typical examples and coding results for the growth stage (partial).

First-order concepts and typical examples cited	Second-order themes	Aggregate dimensions
Complementary advantages “*For so many years, peers are familiar with each other’s advantages… later, some of our orders cannot be produced on time, so we asked our peers to do them. and some of their orders they did not want to do, they would outsource to us to do it*…*” (entrepreneur’s wife)* Cooperative innovation *“Many partners are growing up together with us, and usually take care of us, sometimes we cooperate to bid for some big orders, and some production links, based on feedback from customers and suggestions from peers, we all work together to carry out innovative experiments to improve the process and enhance performance” (entrepreneur)*	Communitarian identity	Entrepreneur’s social identity
Benefit sharing *“Some packaging boxes, accessories and other components are not produced by ourselves now, because these things are much cheaper to buy from the market than to produce ourselves, and they (suppliers) can also make profits.” (entrepreneur)* Information sharing *“They (community members) are also very willing to communicate with us… Especially in the communication with some suppliers and customers, I found out the gap with our peers in the management of raw materials, inventory, quality and other aspects, and absorbed some of their advanced practices to improve our work” (entrepreneur)*		
Balancing short- and long-term goals *“In the short term, the increase in business volume will bring certain profits, but if we blindly pursue the number of orders, in the long run, our technological advantages will be difficult to exert well, which will be detrimental to the long-term development of the enterprise*…*” (entrepreneur)* Value chain horizontal disintegration *“We outsource logistics, accounting, advertising and other businesses, and seek peer OEM for some low-margin and niche orders.” (entrepreneur)*	Broad systematic thinking	Sustainable leadership
Translational skills *“By communicating with my peers and getting some suggestions for improvement, I conducted iterative experiments in the core segment to improve the process* …*” (entrepreneur)*	Innovation and continuous improvement	
Valuing employees *“I did not go to the workshop very often before, but later I paid more attention to this aspect. When I had the opportunity, I went to the workshop to communicate with the employees, to understand their demands and listen to their opinions and suggestions.” (entrepreneur)* Open to suggestions *“During regular company meetings, employee representatives are invited to participate and encouraged to speak, so that employees’ opinions can be listened to. Their opinions are constructive because they have front-line experience (entrepreneur)*	Employees’ engagement	
New market exploration *“With the improved performance of the products and timely delivery, some customers entrust us with their new product requirements, and the market share of some products has increased from the 30 to 70% now” (entrepreneur’s wife)* New product development *“Some customers have asked us to make some product assemblies, and they provide us with bases and copper wires to put the cores, coils and retainers together and tune them according to the parameters required.” (entrepreneur)*	Opportunity seeking	Strategic entrepreneurship
Achieve economies of scale *“Because of the large amount of our commonly used materials, sometimes we can get a little more discount than our peers in terms of price. When the supply is tight, we will be given priority to supply.” (entrepreneur’s wife)* Efficiency improvement *“In the past, there used to be a particularly large number of product types, and we were very slow in delivery and search and often fined for sending the wrong goods, but now it’s much better.” (warehouse manager interview).* Cost control *“Now the probability of mixing material has dropped significantly, reducing the labor cost of the secondary inspection of semi-finished products, and also reduces the unnecessary trouble; raw material procurement is very convenient, and the goods will be sent over as soon as we sent an information.” (entrepreneur’s wife)*	Advantage seeking	

Value chain horizontal disintegration also has an important impact on enterprise’s advantage seeking. First of all, with the increase in the share of core orders, the procurement volume of common materials continues to increase, which allows the company to achieve economies of scale in procurement. It can also reduce logistics and warehousing costs through optimization of procurement frequency and quantity. At the same time, with the improvement of trust relationships among community members and the improvement of the effectiveness of relationship governance and contract governance, many intermediate links are eliminated and transaction costs are reduced.

Secondly, after order optimization, workers do not have to frequently switch back and forth between different types of strips and tools, and the efficiency of gluing, packaging, and clamping has also been greatly improved, so that the articulation and continuity between the links have been improved. This reduces the probability of mixing, and lowers the labor cost of semi-finished product selection and secondary inspection. The improvement of efficiency and the increase in compensation are closely linked, and the well-being of employees is satisfied. The employee’s work-related well-being leads to higher employee productivity and efficiency, which ultimately enhances the company’s competitive advantage and achieves better workplace performance.

This finding also echoes and sublimates the research conclusion of existing research that sustainable leadership, such as amicable labor relations, valuing employees and balancing short-and long-term goals (Suriyankietkaew and Avery, 2016; Awan and Khan, 2021) behaviors can make employees speak up in different ways. At the same time, stakeholders improve community relations through positive and meaningful cooperative behaviors (Iqbal and Piwowar-Sulej, 2022), and ultimately achieve the improvement of overall performance at the individual, organizational and community levels (Iqbal et al., 2018, 2020; Sahai and Mahapatra, 2020; Iqbal and Piwowar-Sulej, 2022) through relationship governance and contractual governance (Awan and Khan, 2021).

The relevant representative materials are cited in Table 5.Therefore, this paper proposes:

**Proposition 2**: In the growth stage, the Communitarian identity of entrepreneur enhances his sustainable leadership, which allows him to choose the path of value chain horizontal disintegrate to implement strategic entrepreneurial behavior.

### Entrepreneur’s communitarian and missionary hybrid identity, SL and SE (the expansion stage: 2016 to date)

#### The formation of communitarian and missionary hybrid identity

Communitarian entrepreneurs usually create products that meet some novel needs of customers in their research domains, and sometimes they also creating new products for their own use because their own needs are not satisfied by existing market products. Hence, their newly developed products often have entirely new functional dimensions, sometimes opening up a new frontier in the industry. The problems solved by creating these new products reflect those needs that the entrepreneur experienced himself, and these needs led to the development of the new product (Fauchart and Gruber, 2011).

Entrepreneurs with a Missionary identity will actively respond to the call of the nation and the concerns of the community. They tend to change the consumption patterns of customers by producing more environmentally friendly and socially responsible products, and contribute to society and the environment. Missionary entrepreneurs believe that firms can act as powerful agents of social change or industrial ecological optimization, and they can build a platform by creating new companies. On this platform, they can pursue their mission visions, advance particular causes, and seek to act in a responsible, transparent and empathetic manner to make the industry ecology and society better (Fauchart and Gruber, 2011).

In 2016, a series of changes in the corporate environment made challenges and opportunities coexist. Challenges were mainly reflected in the supply of raw materials, while opportunities were reflected in the new national entrepreneurial support policies during this period. On the one hand, the entrepreneur and some peers often found that the quality of medium and high-grade strips was unstable during production, which seriously affected the performance of some products. Over the years, the raw material market has been oligopolistic, lacking a perfect bidding mechanism, so the entrepreneur and peers had no bargaining power in procurement. In recent years, strip prices have gradually increased, and the profits of downstream enterprises have been shrinking year by year. These issues put the company under enormous pressure to be sustainable and meet the needs of stakeholders. On the other hand, during this period, mass entrepreneurship and innovation were on the ascendant, and the executive meeting of China State Council established a total scale of 40 billion yuan for emerging industry venture capital guidance funds. Chinese government issued the “Thirteenth Five-Year Comprehensive Work Plan for Energy Conservation and Emission Reduction,” which regards energy conservation and emission reduction as a breakthrough in optimizing the economic structure, promoting green recycling and low-carbon development, and accelerating the construction of ecological civilization. These entrepreneurial incentive policies are a new development opportunity for some high-tech and new energy companies including PX Electronics.

During the communication with the community members, some key customers especially expected the entrepreneur to take effective measures to ensure the reliability of the product performance. Some community members even suggested the entrepreneur to get rid of excessive dependence on the original suppliers, and develop and produce strip materials by himself, so as to fundamentally solve this problem. The entrepreneur also recognized his mission and felt that he had a responsibility to do something to meet the needs of themselves and community members.

Based on this, during this period, the social identity of the entrepreneur gradually evolved into a hybrid identity with the coexistence of Communitarian identity and Missionary identity. The relevant representative materials are cited in Table 6.

**Table 6:** Typical examples and coding results for the expansion stage (partial).

First-order concepts and typical examples cited	Second-order themes	Aggregate dimensions
Responding to community expectations *“Once, a peer said to me: ‘you have the technology and the production conditions, why not try to produce the strip yourself.’ After I came back, I started the relevant experiments*…*” (entrepreneur)* Industry ecology optimization *“There are fewer medium and high-grade strip suppliers, and there is no perfect bidding mechanism. Prices have risen year after year, profit margins have shrunk, and everyone can only passively accept*…*” (entrepreneur)*	Hybrid Identity (Communitarian and missionary)	Entrepreneur’s social identity
Respond to social appeals *“Nanocrystalline soft tape is a new material project, which is in line with local investment promotion policies. If you can apply to settle in the industrial park, you can enjoy policy support and tax incentives in terms of land, energy, and finance.” (entrepreneur)* Energy saving *“In the transportation of magnetic cores, we use recyclable packaging boxes; improve the production process and reduce the emission of pollution” (entrepreneur)*		
Efficient use of resources *“We have improved the process of the heating furnace, optimized the process flow of the upper and lower links, and now the heat energy can be fully utilized, and the power loss has been improved.” (entrepreneur)* Regional economic development *“The local government is satisfied with the environmental protection measures such as sewage, dust and noise in our project application, and is optimistic about the expected benefits of the project and the development of the regional economy”(entrepreneur)*	Corporate social responsibility	Sustainable Leadership
Innovative experiments *“I kept collecting information, observing their (suppliers) process, purchasing raw materials for testing, and using produced strip samples for core production tests… Gradually mastered strip production technology”(entrepreneur)* Performance improvement experiments *“I compared the use of strips with the feedback from customers to find out some common problems as the direction of further improvement and keep improving the product performance”(entrepreneur)* Value chain vertical integration *“In 2016, we extended our technological advantages to the upstream raw material production chain and established a raw material processing enterprise in Shandong to focus on the R&D and production of strips” (entrepreneur)*	Continuous learning and innovation	
Market share expansion *“The relationship between upstream and downstream enterprises in this industry is relatively strong… Customers have a better overall impression of us, not only will they increase their share of purchases, but also introduce other customers and peers to buy your products”(entrepreneur’s wife)* Provision of new services *“We now have two customers asking us to provide product integration services, one for magnetic core assemblies and one for inductor assemblies… The number of new service types and new customers continues to rise.” (entrepreneur)*	Opportunity seeking	Strategic Entrepreneurship
Performance advantage *“At present, the optimal parameters of our products have already reached the performance standards of similar products in Germany… Now the products have entered the procurement catalog of a state-owned enterprise and have begun mass supply.” (entrepreneur)* Improve bargaining power *“In the past, in the procurement of raw materials, we basically passively accepted the price, now the company has more opportunities to know the relevant product prices in the industry. In the market negotiations, we also have more bargaining power”(entrepreneur)*	Advantage seeking	

#### Hybrid identity, sustainable leadership, and value chain vertical integration

Among the hybrid identity of entrepreneur, the Communitarian identity enables them to capture the concerns and demands of community members in a timely manner, and the Missionary identity enhances the entrepreneur’s sense of responsibility. On the one hand, entrepreneurs need to overcome the instability of materials to ensure the stability of product performance, and meet the interests of community members; on the other hand, entrepreneurs also strive to respond to the national call to raise social and environmental awareness. The interaction of the two identities puts forward higher requirements for the SL of entrepreneur, which requires entrepreneur to improve their SL through a series of activities such as continuous learning, community collaboration and innovative behavior.

In order to solve the quality problem of raw materials, entrepreneur took the initiative to conduct strip research and development trials, focused on the study of strip research and development technology, actively communicated with community members to obtain relevant technical information, and carried out research and development experiments with the cooperation of internal staff. After a period of exploration, they basically met the technical requirements for strip production.

“*We look for opportunities to visit the production lines of upstream companies, learn about their processes, carry out experiments in the workshop, trial production with developed strip samples, and get feedback data to improve the experiments*.”*(entrepreneur)*

In the daily production of enterprises, the social and environmental consciousness of the entrepreneur prompted him to actively respond to the national call to enhance corporate social responsibility, improve production processes, optimize efficient use of resources, and reduce energy consumption. Recyclable packaging boxes were used in production, and more environmentally friendly discharge methods were adopted for the company’s sewage, dust and noise to reduce pollution emissions. Meanwhile, the entrepreneur’s responsibility enables him to gain more identification from community members, who are willing to help his innovation activities. This not only helps entrepreneur to quickly grasp the ability of strip R&D, but also provides decision-making reference for their strip production enterprise’s site selection and factory construction. Therefore, after systematic thinking, the entrepreneur made the decision to extend the value chain by transforming skills, upgrading technology, integrating resources and other SL approaches.

In 2016, the entrepreneur obtained investment information from a relative in Shandong. This information is about the investment promotion of Shandong Provincial Government for new energy and new materials innovation and entrepreneurship projects. Nanocrystalline soft magnetic strip material belongs to the new materials project, in line with the local investment promotion policy. If the project can apply to settle in the industrial park, it can enjoy policy support and tax incentives in terms of land, energy, finance, etc. The entrepreneur conducted a systematic evaluation of his raw material R&D project, and decided to apply for the establishment of a factory in Shandong.

“*The power consumption during production is large, and 4 sets of high-power transformers need to be installed to build a factory in Shanghai. The initial installation fee will cost more than 2 million, and other aspects such as land leasing and plant construction are also a big investment in Shanghai*.*” (entrepreneur)*

Entrepreneur actively submitted project applications, and after a series of evaluations, he successfully obtained the admission qualification. In 2016, he chose the strategic entrepreneurial path of vertical integration of the value chain, and established a strip production enterprise CL Electronics in Weifang City, Shandong Province, focusing on the R&D and production of strips. The SL decision of the vertical integration of the value chain enables entrepreneur to meet their own production needs while effectively alleviating the concerns of peers, achieving sales and profit growth, sustainable corporate growth, and enhancing his own industry status. The more relevant representative materials are cited in Table 6.

#### Value chain vertical integration and SE

In the expansion stage, based on the Communitarian and Missionary hybrid identity, through a series of SL behaviors, the entrepreneur made sustainable decisions of the vertical integration of the value chain, which promoted the implementation of corporate SE. In this part, it will discuss the impact of value chain vertical integration, the SL behavior, on the opportunity seeking and advantage seeking of SE.

Value chain vertical integration has a positive impact on the opportunity seeking of the company. Firstly, vertical integration facilitates information sharing by weakening the motivation of knowledge misappropriation and better protecting the possession of information among the upstream and downstream enterprises. This enables PX Electronics to have more rights and channels to collect valid information from its own subsidiary, CL Electronics, instead of collecting information from less closely affiliated suppliers. This information can promote the technological advantages of enterprises to serve new product R&D activities and performance improvement experiments in various ways such as technology coupling and transfer, and promote the opportunity seeking of PX Electronics.

Secondly, the value chain vertical integration allows the expansion of the enterprise value network, enables the enterprise to reach more new customers and markets, helps the entrepreneur find new partners, develop new product marketing strategies and sales channels based on new customer needs and new market criteria, and facilitates opportunity seeking.

In the case of this paper, after the value chain integration, the enterprise continuously conducts performance improvement experiments through technical collaboration between upstream and downstream enterprises. At the same time, the entrepreneur actively seek advice from community members to learn advanced technologies and experiences, which effectively improve product performance through knowledge absorption, technology embedding and other means, and provide more support for product reputation dissemination and new customer acquisition. When CL Electronics was first established, it encountered difficulties in the purchase of accessories and product selection. The thickness of the strip could not be effectively controlled during production, resulting in poor product stability, and due to the poor connection of various processes, the production capacity of the company could not be improved.

“*Because strip production is closely related to high-temperature heating, the requirements for components are very high. As long as there is a problem with one piece, the furnace will be stopped. Later, we actively asked some peers for advice and learned from advanced enterprises. After that, we shared the information we obtained with the employees, and jointly carried out improvement experiments. Finally, the problem of adjusting the distance between the machine and the mold was solved, the quality of the strip was improved, and the raw material demand of the downstream enterprise PX Electronics has been ensured*.*”(entrepreneur)*

At the same time, the entrepreneur compares the feedback from peers on the use of CL Electronics strips with their own experience to identify some common problems as a direction for further improvement. Through this continuous product performance improvement experiment, the product performance was significantly improved at the end of 2019. During the return visit, the entrepreneur said,

*“At present, the optimal parameters of our products have reached the performance standards of similar products in Germany, but unfortunately have not yet been internationally certified, and we have planned to do this certification in the next step. Now the products have entered the corporate procurement directory of a domestic aviation industry, and have begun mass supply.”(entrepreneur)*

Vertical integration of the value chain also has a facilitating effect on the enterprise’s advantage search. First, the vertical integration to the upstream of the value chain based on technological advantages has improved the quality of raw materials and greatly relieved the situation of tight supply of raw materials. By improving the resource creation and control capabilities of enterprises, it can reduce transaction uncertainty and transaction costs, have obvious cost advantages, and also ensure timely supply. Secondly, the vertical integration to the upstream of the value chain reduces the technical barriers and communication barriers between the upstream and downstream, so that the upstream raw material production technology and the midstream product processing technology remain consistent and advanced, so that technological advantages can be quickly converted into commercial value.

The case code shows that the creation and production of CL Electronics has enabled PX Electronics to have more choices and autonomy in the selection of strips. “*The strips in Shandong can be delivered as needed without occupying the expensive storage space in Shanghai,”* which can reduce storage and logistics costs. At the same time, as there was no trust worry between upstream and downstream enterprises, the coordination efficiency was improved, and the communication cost and transaction costs were reduced. Moreover, upstream and downstream enterprises can not only share technologically advantageous resources, but also share costs in sales, advertising, marketing, etc., which allows the enterprise to gain cost advantages. There are certain strategic support advantages between upstream and downstream enterprises, which also enhances the industry status and market competitiveness of enterprises.

Through the analysis of qualitative materials, it can be found that in this stage, the founder actively responded to community concerns, enhanced social responsibility, completed vertical extension of the value chain through sustainable leadership behaviors such as deep learning and skill transformation, developed and produced high-quality strips, and alleviated the procurement dilemma faced by community members. This finding also echoes and sublimates the research conclusion of existing research that sustainable leadership, such as long-term perspective, corporate social responsibility (Avery and Bergsteiner, 2011), systemic innovation (Avery, 2005; Iqbal et al., 2020), can promote creative problem-solving skills and deep learning (Wolff, 2020), etc., helps business managers balance short and long-term interests, and obtain overall benefits and sustainable growth at individual, company, and community levels. This case evidence also presents the foundation for future studies and a bridge associating prior research.

The relevant representative materials are cited in Table 6. Based on the above analysis, we propose the following propositions:

**Proposition 3**: In the expansion stage, the hybrid identity of entrepreneur enhances his sustainable leadership, which allows him to choose the path of value chain vertical integration to implement strategic entrepreneurial behavior.

## Conclusion and discussion

### Conclusion

This case evidence presents the foundation for future studies and a bridge associating prior research. Based on entrepreneurial identity theory and SL theory, this paper explores the path selection and behavioral mechanism of SE in technology-based family firms from the perspective of the evolution of entrepreneurial social identity. Particularly, this study explores and identifies the mediating effect of SL on the relationship between the social identity of the entrepreneur and SE. It promotes the application of SL in the strategic entrepreneurial activities of family businesses, and expands the research context of SL. Thus, the research provides theoretical basis and action guidelines for family firms to effectively cope with risks and challenges, to achieve wealth creation and sustainable growth in volatile economic times.

The case study found that at different stages of SE of technology-based family firms, entrepreneurs improved their own SL through the dynamic adjustment of their social identity types. This leadership enhancement enables entrepreneurs to carry out value chain disintegration and integration activities through the application, focus and extension of technological advantages. By doing so, entrepreneurs are able to advance the implementation of the company’s SE, and promote the sustainability of the company.

During the entrepreneurial planning stage, the entrepreneur identified entrepreneurial opportunities based on previous experience and self-evaluation. Through continuous learning and technology application, entrepreneurs actively built a legal and unique entrepreneurial identity, and completed the transition from employee identity to entrepreneur identity, which laid the foundation for the development of entrepreneurial activities.

In the early stage of entrepreneurship, due to the pressure of survival and highly uncertain resource constraints, entrepreneurs present a Darwinian social identity. The strategic entrepreneurial behavior and path chosen by the entrepreneur in this phase is resource acquisition. The entrepreneur acquires resource support from internal and external stakeholders through appropriate identity narratives and sustainable leadership approaches to facilitate the identification of entrepreneurial opportunities and the acquisition of competitive advantage, which in turn facilitates the implementation of strategic entrepreneurship and enables the firm to acquire sustainable growth. The main entrepreneurial motivation during this period was the creation of profitable enterprises to maximize economic benefits. Therefore, based on their own technological advantages, entrepreneurs, on the one hand, are driven by their vision to obtain entrepreneurial support from their families and attract like-minded people to form entrepreneurial teams. On the other hand, based on common interests, entrepreneurs actively seek external stakeholders to obtain identification and resource support. By organically integrating the resource support from stakeholders with their own technology transformation capabilities, entrepreneurs can quickly complete the creation of their businesses and gain profits through a series of SL behaviors such as technology application, innovative cooperation models and rapid integration of resources.

In the growth stage, with the increase in business transactions, entrepreneurs and community members have more interest connections and symbiotic relationships, so the social identity of entrepreneur evolves into a Communitarian identity. In this stage, the strategic entrepreneurial behavior and path chosen by the entrepreneur is the value chain horizontal disintegrate. By outsourcing some non-core businesses, entrepreneurs focus on core businesses that leverage their technological strengths. Communitarian identity helps the entrepreneur gain the trust and support of external stakeholders. Long-term cooperation promotes the complementarity and division of labor among community members. This is because after the accumulation in the early stage of entrepreneurship, the foundation of mutually beneficial transactions between enterprises and community members has been formed, and a more standardized market transaction method has emerged, which provides more possibilities for cooperation among community members. Based on this situation and changes in the external environment, entrepreneurs, through systematic thinking, innovation and continuous improvement, carry out SL behaviors such as division of labor and complementary advantages among members. These behaviors are likely to allow the entrepreneurs to divest redundant resources and highlight technological advantages through the strategic entrepreneurial path of value chain horizontal disintegration, which helps enterprises to obtain innovation opportunities and competitive advantages and achieve sustainable growth.

During the expansion stage, entrepreneurs’ social identities presented a hybrid identity of Communitarian and Missionary. The strategic entrepreneurial behavior and path chosen by entrepreneurs in this phase is the vertical integration of the value chain. By expanding the application of technological advantages, the entrepreneur extends the value chain to the upstream raw material research and development link, enhancing the resilience of the enterprise’s raw material supply and its own industry competitiveness. During this period, on the one hand, the entrepreneur actively responded to the national call, paid attention to environmental protection and social benefits, and actively carried out energy conservation and emission reduction and green innovation activities; on the other hand, the entrepreneur actively responded to community concerns and raised his sense of responsibility. By utilizing the technological advantages to R&D strip materials, he helped community members effectively deal with the dilemma of raw material procurement. The combination of the two identities enables entrepreneurs to continuously improve their SL through continuous learning, transitional skills, collaborative innovation and other activities. This prompts them to integrate external resources and expand their technological advantages through the strategic entrepreneurial path of vertical integration in the value chain, which enables them to search for entrepreneurial opportunities and competitive advantages.

The findings of this paper suggest that the entrepreneur’s subjective initiative and the multilevel identity of the entrepreneur play an important role in the SE process of technology-based family firms. Entrepreneurs can adjust the salience of different social identity types based on changes in the entrepreneurial context, and carry out SL behaviors through the evolution of social identities, thereby promoting the implementation of SE in the business.

The research finding also suggests that technology-based family firms can choose appropriate strategic entrepreneurial paths at different stages of entrepreneurship through SL approaches such as focusing and extending the technological advantages, with the goal of entrepreneurial opportunity seeking and strategic advantage seeking, to ultimately achieve value creation and sustainable development of the firm. The findings of this paper provide a new explanation for the choice of strategic entrepreneurial paths for technology-based family firms and bring new insights into the sustainable development of such family firms.

In particular, this study has employed sustainable leadership theory to link the social identity of the entrepreneur with strategic entrepreneurship. It applies SL to the study of strategic entrepreneurship in family businesses, expanding the research context of sustainable leadership theory. The research finds that the SL of entrepreneurs plays an important role in the implementation of firms’ strategic entrepreneurial activities. The study also expands the application of SL in family firms entrepreneurial activities and explores the triggers of sustainable leadership at different stages of entrepreneurship, which responds to the call for in-depth research on SL by scholars such as Burawat (2019), Hallinger and Suriyankietkaew (2018), and Iqbal et al. (2018, 2020, 2021), and expands the research related to SL behavior.

### Theoretical contribution

Existing studies have formed valuable research results on entrepreneurial identity, SL, and family firm SE. Based on these studies, the marginal contributions of this paper mainly include the following aspects:

First, this study provides a new explanatory framework for the path selection mechanism of SE in family firms. The study on SE in family firms have been discussed from the perspectives of resource orchestration (Chirico et al., 2011), inter-generational succession (Lee et al., 2019), family involvement (Bendig et al., 2020), internationalization strategy (Arregle et al., 2017; Zahra, 2020) and so on. Through the literature review, it is found that SE has a positive impact on the performance, strategic change, transformation, upgrading and sustained growth of family firms. However, the implementation paths and behavioral mechanisms of SE in family firms have not been thoroughly explored, which may make it difficult for existing theories to provide effective and clear action guidance for SE in family firms, and firms’ managers do not know how to promote their SE at different stages. Based on the social identity theory of entrepreneurs (Fauchart and Gruber, 2011; Powell and Baker, 2014; Wry and York, 2019), this paper follows the logical paradigm of “antecedent-behavior-outcome” and constructs a strategic entrepreneurial path model for technology-based family businesses from the perspective of dynamic identity evolution. The mechanism of strategic entrepreneurial path selection and behavioral mechanism of technology-based family firms in different entrepreneurial contexts are explained. By doing so, it bridges the gap of existing studies on strategic entrepreneurial paths of family firms and provides a theoretical framework for future empirical research and theory development.

Secondly, this study responds to the call for in-depth research on SL by scholars such as Burawat (2019), Hallinger and Suriyankietkaew (2018), and Iqbal et al. (2018, 2020, 2021), and expands the research related to SL behavior. This study finds that the SL of entrepreneurs plays an important role in the implementation of firms’ strategic entrepreneurial activities, and expands the application of SL in family firms entrepreneurial activities. The research also found that entrepreneurs can improve their SL through activities such as differentiated perception, value chain management, continuous learning and resource orchestration, which help firms perceive opportunities, acquire and construct internal and external resource in dynamic situations. Therefore, this study expands the application of SL in family firms wealth creation and sustainable growth, conducts an extended analysis of SL behaviors, and deepens the theoretical connotation of SL.

Furthermore, this paper enriches the research on the entrepreneurial social identity literature. This study responds to scholars’ calls for research on the multiplicity and dynamics of entrepreneurial identity (Powell and Baker, 2014, 2017; Pan et al., 2019; Mmbaga et al., 2020), clarifies the dynamic evolution of entrepreneurial social identity with changes in entrepreneurial contexts, and explores the impact mechanisms of the evolution of entrepreneurial social identity on entrepreneurial behavior, which expands relevant research on entrepreneurial identity theory, and also provides a useful exploration of the subjective motivation of entrepreneurs in SE.

### Managerial implications

This article can provide managerial implications for wealth creation and sustainable growth of family firms. First, this study finds that with the context changing, entrepreneurs should timely adjust the salience of various social identity types, this identity dynamics affects their strategic decisions and entrepreneurial behaviors.

Therefore, for entrepreneurs, it is important to manage their entrepreneurial identity in different stages, dynamically adjust the salience of every identity, adopt effective management approaches to carry out entrepreneurial activities (such as SL), in order to achieve wealth creation and sustainable growth of the enterprise. In the entrepreneurial planning stage, entrepreneurs should systematically think about their own advantages, the opportunity traits and industry characteristics, choose the domains that can leverage their advantages for entrepreneurship, and actively build a legitimately distinctive entrepreneurial identity. In the initial stage, entrepreneurs can focus on entrepreneurial resource acquisition, team building, and opportunity identification based on Darwinian social identity, and strive for identification and resource support from more potential stakeholders with shared vision and interest claims, so that the enterprise can gain entrepreneurial legitimacy and enter the market smoothly and obtain economic benefits quickly. In the growth stage, entrepreneurs can focus on their own advantageous domains through the division of labor and complementarity among community members based on Communitarian identity, continue to carry out iterative experiments, seek to improve product performance, upgrade technological advantages, and optimize the allocation of key resources, in order to promote the enterprise’s opportunity seeking and advantage seeking. During the expansion stage, entrepreneurs can seek diversified development and promote the implementation of SE through vertical integration of the value chain and expansion of the advantageous areas based on the Communitarian and Missionary hybrid identities or other types of identity.

Second, the mediating role of SL in the relationship between entrepreneurial identity and SE suggests that in practice, entrepreneurs should be able to choose SL behaviors that match the entrepreneurial opportunity seeking and competitive advantage seeking according to specific periods and situational changes. In this way, it can achieve resource acquisition and effective allocation to avoid risks, obtain stable returns and sustainable competitive advantages.

Third, for policy makers, when formulating supportive policies related to entrepreneurship, they should not only consider factors such as products, technologies and markets of entrepreneurial enterprises, but also should pay more attentions to the construction of the institutional environment. It is necessary to consider the development stage of entrepreneurial enterprises, especially the identity characteristics of entrepreneurs, so as to introduce more targeted financial and tax policies. Through active policy guidance and incentives, it is possible to promote technological upgrading, technological transformation, reform and innovation of entrepreneurial enterprises to achieve sustainable and healthy development of the industry.

### Limitations and future research

Despite the abovementioned contribution, this study has several limitations that open new research opportunities. First of all, this paper adopted a single case study, so the external validity of the proposed theoretical proposition and model needs to be further tested. In the future, multiple case studies or a statistical large-sample empirical research ought to be conducted to improve the proposition and further verify the validity of the conclusion; Secondly, this study only discusses the role of mediating variables and does not consider the moderating effect. Future research ought to consider the moderating effects of contextual factors such as environmental dynamics, resource constraints, and the stability of interest linkages between stakeholders. Furthermore, this study chose technology-based family business as the research object. Whether the conclusions are valid for other types of enterprises also needs further research. In the future, cross-industry research can be conducted to improve the applicability of the research conclusions.

## Data availability statement

The original contributions presented in the study are included in the article/supplementary material, further inquiries can be directed to the corresponding author.

## Author contributions

GL and QY developed the research project, conducted the field study, and reviewed the literature. QY, GL, and LZ carried out the data analysis and reviewed and edited the manuscript. All authors contributed to the article and approved the submitted version.

## Funding

This research was funded by the National Social Science Foundation of China (no. 17BGL030).

## Conflict of interest

The authors declare that the research was conducted in the absence of any commercial or financial relationships that could be construed as a potential conflict of interest.

## Publisher’s note

All claims expressed in this article are solely those of the authors and do not necessarily represent those of their affiliated organizations, or those of the publisher, the editors and the reviewers. Any product that may be evaluated in this article, or claim that may be made by its manufacturer, is not guaranteed or endorsed by the publisher.
